# Meta-analysis of Proton Pump Inhibitors in the Treatment of Pharyngeal Reflux Disease

**DOI:** 10.1155/2022/9105814

**Published:** 2022-07-21

**Authors:** Xiulin Jin, Xufeng Zhou, Zongxian Fan, Yingchun Qin, Junjie Zhan

**Affiliations:** Department of Otorhinolaryngology, First Affiliated Hospital of Jiamusi University, Jiamusi City, Heilongjiang Province, China

## Abstract

The present study aimed to examine the safety and healing effects of proton pump inhibitors (PPIs) in people with laryngopharyngeal reflux disease (LPRD). To find all relevant studies published before April 1, 2022, we searched the PubMed, Embase, Web of Science, Clinical Trials, Cochrane Library, CNKI, and Wanfang databases. For SLE, we looked for all randomized controlled clinical trials related to PPIs versus placebo-controlled treatment of LPRD. Overall efficiency, reflux symptom index (RSI), reflux finding score (RFS), improvement in cough and hoarseness, and adverse reactions were compared using the Review Manager 5.3. Using the reflux symptom index (RSI) as an outcome indicator for efficacy assessment, the PPI group showed significant improvement compared with the placebo group [MD = 3.35, 95% CI (1.34, 5.37, *P* < 0.05)]. In terms of overall efficacy, the PPI group showed effectiveness, but its efficacy was not statistically significantly dissimilar from that of the placebo group [OR = 1.62, 95% CI (0.89, 2.95), *P* > 0.05].

## 1. Introduction

Laryngopharyngeal reflux disease (LPRD) is a term used to describe a variety of symptoms and signs brought on by the reflux of stomach contents into the pharynx through the upper esophageal sphincter (UES) [1]. Due mostly to mucosal irritation that causes an inflammatory response and excessive mucus secretion, LPRD is currently regarded as one of the most prevalent chronic inflammatory disorders of the upper respiratory tract [2]. Clinical symptoms include foreign body sensation in the throat, persistent throat clearing, hoarseness, chronic cough, and laryngeal signs such as mucous membrane hyperplasia and hypertrophy in the posterior vocal fold area, diffuse congestion, and edema of the vocal folds [3]. In recent years, there has been a gradual increase in the number of patients with chronic, nonspecific throat discomfort associated with reflux seen in otolaryngology. Epidemiological surveys have found that the prevalence of LPRD in otolaryngology outpatients is 10% [4], European data show that the prevalence of LPRD is about 18.8% [5], while domestic surveys have found that the prevalence of LPRD is about 5% [6].

The etiology of LPRD is not well understood, and some studies have reported mechanisms associated with LPRD: direct contact between gastroesophageal reflux and the pharyngeal mucosa, acid stimulation of the vagus nerve, and lack of resistance of the pharyngeal mucosa to gastric acid compared to the esophageal mucosa [7, 8]. Small amounts of acid may not be sufficient to cause esophageal symptoms but may be sufficient to cause throat symptoms. Pharmacological intervention with PPIs, lifestyle changes, and dietary modification are now recommended as treatment strategies for LPRD [9]. PPIs are commonly used in the clinical empirical treatment of laryngopharyngeal reflux diseases. Inhibiting H + -K+ -ATPase on gastric wall cells, decreasing gastric acid output, decreasing pepsin activity, and blocking the inflammatory response are the treatment methods used to lessen the direct throat damage [10]. However, the effectiveness of proton pump inhibitors in the treatment of laryngopharyngeal reflux disease has long been controversial. The efficacy and safety of PPIs in the treatment of patients with LPRD remain controversial, and further exploration of the efficacy and safety of PPIs in the treatment of LPRD is therefore warranted.

The efficacy and safety of PPIs are still controversial, and there is no standardized treatment protocol. Therefore, this meta-analysis aims to further investigate the therapeutic effects and safety of PPIs in LPRD.

The rest of the article is as follows: Section 2 defines the various methods.  Section 3 evaluates the results.  Section 4 discusses the discussion.  Section 5 concludes the article.

## 2. Methods

### 2.1. Literature Search Strategy

The published literature on PPIs for the treatment of LPRD was located using a computer-based search of the PubMed, Embase, Web of Science, Clinical Trials, Cochrane Library, CNKI, and Wanfang databases. The search period was from the creation of the database until 1 April 2022. English and Chinese are the search languages. Search terms are as follows: “proton pumps antagonists” or “proton pumps inhibitors” or “histamine H2 antagonists” or rabeprazole or esomeprazole or pantoprazole or lansoprazole or omeprazole; laryngitis or pharyngitis or “laryngopharyngeal reflux”(LPR) or “gastro pharyngeal reflux”(GPR); “Randomized controlled trial” or “RCT.”

### 2.2. Eligibility Criteria

The following PICOS criteria were used to cover the studies.

#### 2.2.1. Participants of Various Types

Adult patients aged >18 years with a diagnosis of LPRD-related disease were included in the study.

#### 2.2.2. Interventions

The intervention was PPIs in the experimental group and placebo in the control group.

#### 2.2.3. Types of Result Measures

The primary outcome measures covered the overall efficiency, reflux symptom index (RSI) [11], reflux finding score (RFS) [12], improvement in cough and hoarseness, and adverse reactions.

#### 2.2.4. Types of Studies

Based on inclusion criteria for qualifying trials, full publications and data from randomised controlled studies of PPIs in patients with LPRD were obtained.

The literature was studied individually by two investigators, with the initial screening consisting of reading the abstracts and titles and saving the relevant material that met the inclusion criteria for rescreening.

### 2.3. Information Extraction

According to the proposed criteria, researchers independently extracted data and relevant information from the included literature and recorded the findings, which included the source of the literature (author, date of publication, and country), basic characteristics of the study population (sample size and age), and interventions (type of PPIs and duration of dose study). Researchers must evaluate one another, and if there is a disagreement, a third-party decision is required.

### 2.4. Quality Assessment

Use the Cochrane 5.1 manual's risk of the bias assessment tool to assess the risk of bias in RCT studies [13]. The experimental PPI group was demonstrated to be beneficial overall; however, there was no statistically significant difference between them and the control group.

### 2.5. Statistical Analysis

A meta-analysis of the data was performed using Review Manager (RevMan) 5.3 software. The dichotomous variables (overall efficiency and adverse effects) were expressed as odds ratios, whereas the continuous variables (RSI, RFS, improvement of cough, and hoarseness) were reported as mean differences (OR). Both variables are described using a 95% confidence interval (CI). The included studies were tested for heterogeneity, and a fixed-effects model was used for meta-analysis if I2 was <50%, and a random-effects model was used for meta-analysis if I2 was ≥50%. Studies were considered to be statistically significant if *P* < 0.05. When the number of included studies was greater than or equal to 10, a funnel plot was used for publication bias analysis.

## 3. Results

### 3.1. General Information on the Included Literature

As shown in Figure 1, a total of 4168 relevant articles (72 from CNKI, 92 from Wanfang, 57 from CBM, 47 from Wipe, 88 from Cochrane, 2447 from PubMed, 1029 from Embase, and 336 from Web of Science) were identified according to the search strategy. Cochrane 88, PubMed 2447, Embase 1029, Web of science 336, computerized deduplication of 448 (72 in Chinese and 376 in English), exclusion of 3665 after reading the title abstracts, and further screening of 55 (30 in Chinese and 25 in English) might meet the inclusion criteria by reading the full text. A total of 14 randomized controlled trials that met the exclusion criteria were included.

### 3.2. Basic Characteristics

Fourteen randomized controlled trials included 815 patients with LPR, most diagnosed by laryngoscopy or esophageal pH monitoring, and the 14 studies were conducted in different parts of the world [14–27]. All 14 included papers gave baseline data for the experimental and control groups, which were similar and comparable between the two groups at baseline.  Table 1 summarizes 14 studies with basic information.

### 3.3. Quality Assessment

Of the 14 included studies, one was a crossover controlled trial [21], and the rest were all randomized measured trials. 10 of the studies [14, 15, 17, 20, 22, 23, 25, 27] explicitly stated the method of generating the randomized sequence, and three studies [16, 24, 26] only suggested to randomize patients into experimental and control groups but did not state the method of generating the randomized sequence. The included studies were double-blinded except for the Chappity et al.'s [14] study which was single-blinded to the treatment group; 10 studies [15–20, 22, 23, 25, 26] explicitly gave allocation concealment schemes, and all trials did not selectively report outcomes; 3 studies [20, 22, 23] had missed visits, but the final data analysis excluded those who were missed and the number of people who fully performed the trial procedure for the quasi-analysis, and the remaining outcome data were reported in full (Figure 2).

### 3.4. Meta-analysis Results

#### 3.4.1. RSI Score

Four studies [15, 17, 18, 22] reported a comparison of the improvement in pharyngeal RSI scores before and after treatment in patients with LPRD in the PPIs treatment group, with 132 cases in the experimental group and 105 cases in the control group, with the experimental group outperforming the control group in terms of improvement in RSI scores, with statistically significant differences [MD = 3.35, 95% CI (1.34, 5.37, *P* < 0.05)] (Figure 3).

#### 3.4.2. Overall Efficiency

Ten studies [14, 16, 19, 26] compared the general effectiveness of PPI in patients with LPRD, with 329 cases in the experimental group and 271 in the control group. The outcomes demonstrated that the experimental group was successful; however, there was no statistically significant difference between the experimental group and the control group [OR = 1.62, 95% CI (0.89, 2.95), *P* > 0.05] (Figure 4).

#### 3.4.3. RFS

Four studies [15, 17, 18, 22] reported a comparison of PPI on pharyngeal RFS scores in patients with LPRD, with 112 cases in the experimental group and 105 cases in the control group, with no statistical difference in RFS scores [MD = 0.62, 95% CI (-1.28, 2.48), *P* > 0.05] (Figure 5).

#### 3.4.4. Improvement of Cough and Hoarseness Symptoms

Seven studies [15–18, 22, 24, 27] compared the improvement of PPI on cough in patients with LPRD, including 159 cases in the experimental group and 144 cases in the control group. There was no difference in the rate of relief of cough symptoms in patients with LPRD by PPI compared with the control group, and there was a strong placebo effect [SMD = −0.12, 95% CI (-1.44, 1.19), *P* > 0.05] (Figure 6). Five studies [16–18, 22, 24] compared the improvement of hoarseness in patients with LPRD by PPI, with 129 cases in the treatment group and 119 cases in the control group, with no statistically significant difference between the two groups in terms of relief of hoarseness symptoms [SMD = −0.51, 95% CI (-1.36, 0.35), *P* > 0.05] (Figure 7).

#### 3.4.5. Adverse Effects

The results of the meta-analysis could not be combined due to inadequate reporting of data on adverse reactions in the included studies. We only performed descriptive analyses. 2 studies explored adverse reactions, and the results of Shaheen et al. [15] showed that no serious adverse drug reactions occurred during dosing and no patients withdrew from the study due to the safety of the drug. Vaezi et al. [20] showed that the experimental group experienced increased upper respiratory tract infections and discomfort with monitoring medical devices and gastrointestinal reactions compared to the control group; a higher proportion of patients in the experimental group experienced increased upper respiratory infections and discomfort and gastrointestinal reactions to monitoring equipment compared to the control group. There were no significant changes in weight, changes in vital signs, or relevant ECG parameters in either group, and there was a trend towards increased gastrin levels in the experimental group.

## 4. Discussion

Laryngopharyngeal reflux is a chronic inflammatory disease with no clear cause, which explains why it is so simple to misdiagnose given that its clinical symptoms are similar to those of many other laryngopharyngeal diseases. The RSI and RFS score scales are primarily used to screen patients for diseases by precisely assessing their clinical symptoms and indicators [28]. Changes in pepsin levels, gastric bubble size, and laryngopharyngeal reflux disease are somewhat correlated [29, 30]. A sore throat and hoarseness are relatively obvious symptoms of this disease. Symptoms such as persistent coughs, foreign bodies in the throat, and shortness of breath seriously impact patients' feature of life. Vocal cord edema is accompanied by glottis stenosis, mesangial hyperplasia, granulomas, diffuse congestion, and glottal stenosis. Laryngitis and pharyngitis can cause serious health problems, including chronic laryngitis and pharyngitis which negatively impact patients' physical and mental health if not treated promptly and effectively [31]. To promote a good prognosis and recovery for patients suffering from laryngopharyngeal reflux disease, rapid diagnosis and effective treatment are very important [32].

Proton pump inhibitors are commonly used in the clinical empirical treatment of laryngopharyngeal reflux diseases. It works by inhibiting H + -K+ -ATPase on the gastric wall cells, reducing the excretion of gastric acid, reducing pepsin activity, and reducing inflammation, thereby reducing the effects of direct damage to the throat [33]. In clinical practice, many practitioners recommend the use of PPIs to improve symptoms associated with patients with LPRD and consider them to be effective. However, the effectiveness of proton pump inhibitors in the treatment of laryngopharyngeal reflux disease has long been controversial. In a study by Gatta et al. [34], there was no discernible improvement in reflux symptoms between PPIs and placebos. The reasonable use of PPI is a more successful treatment for GERD pharyngitis, according to a domestic meta-analysis conducted by Zhang et al. in 2012 [35], and this discrepancy in the results has significantly impacted the marketing of this medication. Therefore, there is a need for a comprehensive evaluation of the efficacy of proton pump inhibitors in patients with laryngopharyngeal reflux disease through evidence-based medicine to provide a reliable evidence-based basis for the treatment of laryngopharyngeal reflux disease.

In the RSI score, the experimental PPI group was better than the control group in comparing the RSI score of throat symptom improvement, and the efficacy was statistically significant, and the difference between the two was statistically significant. The throat symptoms such as foreign body sensation in the throat and persistent throat clearing in the PPI treatment group improved significantly, which can be used as a reference to guide the clinical use of drugs. The mechanism of the improvement of throat symptom improvement by PPI is that PPI inhibits the H + - K-- ATPase, which reduces gastric acid secretion and pepsin activity, thereby reducing the direct damage to the throat. Five of the 13 randomized controlled trials that included 831 patients with LPRD in Wei, which used the RSI as an outcome indicator to assess the efficacy of PPI, showed significantly better improvement in RSI scores in the experimental group than in the placebo control group [36]. However, Liu et al. [37] included eight studies containing 370 patients in their 2016 meta-analysis, which showed a nonsignificant efficacy of the experimental group compared to the control group in terms of overall efficiency and improvement in cough symptoms in patients with LPRD. The difference in results compared to our study may be due to the relatively high quality of the included studies due to our inclusion of larger sample size and the development of strict inclusion and exclusion criteria. However, as the RSI does not cover all symptoms and should be used in conjunction with patient symptom improvement as an indicator of efficacy assessment, it is expected that subsequent studies will provide more objective indicators to evaluate the efficacy of PPI for LPRD.

In terms of overall effectiveness, the experimental PPI group was shown to be effective, but the difference with the control group was not statistically significant. We speculate that this may be due to the variability in lifestyle and diet of patients with LPRD. The expert consensus on LRPD states [38] that changing poor lifestyle and diet is the most basic treatment strategy, but the guidelines do not specify specific dietary interventions. Traditional dietary interventions suggest reducing the intake of some acidic foods such as caffeine, beer, and chocolate and using alkaline water, as well as changing lifestyle habits such as the traditional dietary interventions which include reducing the intake of acidic foods such as caffeine, beer, and chocolate and using alkaline water, as well as lifestyle changes such as smoking and alcohol cessation. While clinicians often give verbal advice on the importance of dietary modification in the treatment of LPRD, few studies provide detailed statistics on patient adherence. It is this wide variation in dietary habits that can affect the efficacy of PPI.

PPI did not show significant efficacy in improving RFS scores in adult LPRD patients. RFS is an eight-item grading scale, but it is subjective because the laryngologist who grades it is based on their experience. It has not been proven to be a reliable method for detecting reflux-induced laryngopharyngeal symptoms. Furthermore, because of a lack of standardization and clarification of nomenclature, there was a great deal of diversity in the interpretation of the larynx by both ENT and GI professionals [39].

In adults with LPRD, there is inadequate data to show that PPI has a meaningful benefit over placebo in reducing pharyngeal symptoms including cough and hoarseness. In their study, Lechien et al. noted that dietary changes and lifestyle modifications combined with the use of twice daily pantoprazole showed significant improvement in the symptoms of hoarseness caused by gastroesophageal reflux [40]. However, Johnson et al. applied acoustic parameters as an objective method to evaluate hoarseness and suggested that clinically cured patients (RSI <13 and RFS <7) showed no or little improvement in acoustic parameters and that their study could not confirm whether the significant improvement in voice quality was due to dietary modifications or to the therapeutic effect of PPIs [41]. In a study by Lechien et al., it was noted that esophageal reflux was a cause of chronic cough in adults, that PPI treatment alone was ineffective and had a strong placebo effect, and that lifestyle modification combined with weight loss was beneficial for the improvement of cough symptoms [42]. The efficacy of PPI on cough and hoarseness remains controversial and may be related to the small number of studies included and the inadequate sample size, and it is expected that large sample size and multicenter randomized controlled clinical study will be available in the future to assess the efficacy of PPI on cough and hoarseness. The efficacy of PPI on cough and hoarseness is expected to be evaluated in future large sample size and multicenter randomized controlled studies.

After discontinuation of PPI, more than 90% of patients have a recurrence of symptoms and need to be treated with PPI again, while long-term PPI use has been associated with adverse effects such as reduced calcium and vitamin B12 absorption, increased risk of pulmonary infection, and cardiovascular events [43]. The data on adverse effects in our studies [15, 20] were inadequately reported, and more studies focusing on the safety of PPIs for LPRD are expected at a later stage.

Limitations of this paper are as follows:

- The effectiveness of the drug was evaluated along with adverse drug reactions, but there are too few relevant data reported, so this study was not analyzed for comparison
- Although the criteria for determining efficacy were developed after reading the literature to reduce the heterogeneity of the data, there may be some risk of bias as the meta-analysis is a nonexperimental study, and it is not possible for all included study results to meet the effect indicators

In summary, PPIs were useful in alleviating throat symptoms in LPRD patients but were ineffective in reducing symptoms of cough and hoarseness. It is anticipated that more clinical trials will be conducted in the future to overcome the current limitations by utilizing large samples and multicenter randomized controlled trials with strict and uniform diagnostic and efficacy criteria to determine the true efficacy of PPI on LPRD. Nevertheless, this study still has some limitations, and these limitations will need to be addressed. It is expected that more clinical trials will be conducted in the future to overcome the current limitations, adopt large samples and multicenter randomized controlled trials, conduct rigorous and uniform diagnostic criteria and efficacy assessment to evaluate the true efficacy of PPIs on LPRD, avoid overdiagnosis and treatment, clarify the safety of the drugs, and reduce their side effects.

## 5. Conclusions

PPIs are effective in successful symptoms in patients with pharyngeal reflux disease and are recommended in the treatment strategy for patients with LPRD, possibly in combination with lifestyle alteration.

## Figures and Tables

**Figure 1:** Flow chart of literature search and study selection.

**Figure 2:** Bias risk assessment results included RCT.

**Figure 3:** Comparison of reflux symptom index scores between the experimental group and the control group.

**Figure 4:** Comparison of the overall efficiency of the experimental group and the control group.

**Figure 5:** Comparison of reflux symptom scores between the experimental group and the control group.

**Figure 6:** Comparison between the experimental group and the control group on the relief of cough symptoms in patients with pharyngeal reflux disease.

**Figure 7:** Comparison of the relief of hoarseness in patients with pharyngeal reflux disease between the experimental group and the control group.

**Table 1:** Characteristics of individual studies included in the meta-analysis.

Study (year)	Country	Age (E/C)	Sample (E/C)	Interventions (E/C)	Follow-up (week)	Outcomes
Chappity et al. (2014) [14]	India	36.9	117/117	Omeprazole 20 mg (2 times/d)/lifestyle change treatment only	12	②
Shaheen et al. (2010) [15]	United States	49.5 ± 12/51.0 ± 11.6	22/18	Esomeprazole 40 mg (2 times/d)/placebo	12	①③④⑥
Fass et al. (2009) [16]	United States	63.25 ± 13.33/67.71 ± 9.47	24/17	Esomeprazole 20 mg (2 times/d)/placebo	12	②④⑤
Lam et al. (2010) [17]	China	46.29 ± 9.77/47.43 ± 8.66	42/40	Rabeprazole 20 mg (2 times/d)/placebo	12	①③④⑤
Reichel et al. (2008) [18]	United Kingdom	49 ± 13.9/47.6 ± 16	30/28	Esomeprazole 20 mg (2 times/d)/placebo	12	①③④⑤
Wo et al. (2005) [19]	United States	39/37	20/19	Pantoprazole 40 mg(1 time/d)/placebo	12	②
Vaezi et al. (2006) [20]	Australia	51.5 ± 15.2/50.5 ± 14.5	95/50	Esomeprazole 40 mg (2 times/d)/placebo	16	②⑥
Eherer et al. (2003) [21]	United States	48	10/10	Pantoprazole 40 mg (2 times/d)/placebo	12	②⑥
Steward et al. (2004) [22]	United States	45.8 ± 11.2/52.8 ± 11.5	21/21	Rabeprazole 20 mg (2 times/d)/placebo	8	①②③④⑤
El-Serag et al. (2001) [23]	United States	59/65	12/10	Lansoprazole 30 mg (2 times/d)/placebo	12	②
Noordzij et al. (2001) [24]	United States	51.7/45.3	15/15	Omeprazole 40 mg (2 times/d)/placebo	8	②④⑤
Ours et al. (1999) [25]	United States	54	8/9	Omeprazole 40 mg (2 times/d)/placebo	12	②
Langevin and Ngo (2001) [26]	Canada	53	14/16	Omeprazole 40 mg (2 times/d)/placebo	12	②
Rabeneck et al. (1999) [27]	Australia	54	8/7	Lansoprazole 30 mg (2 times/d)/placebo	12	④

① RSI score; ② overall effectiveness rate; ③ antifluid sign score; ④ relief of cough symptoms; ⑤ relief of hoarseness symptoms; ⑥ adverse effects rate.

## Data Availability

Data to support the findings of this study is available on reasonable request from the corresponding author.
